# Role of alternative splicing of VEGF-A in the development of atherosclerosis

This article has been retracted.

**DOI:** 10.18632/aging.101580

**Published:** 2018-10-13

**Authors:** Naishi Zhao, Jianfeng Zhang

**Affiliations:** 1 Department of Cardiovascular Surgery, Shanghai Chest Hospital, Shanghai Jiao Tong University, Shanghai 200030, China

**Keywords:** atherosclerosis (AS), macrophage, endothelial cells, SRPK1, alternative splicing of VEGF, ApoE (-/-), high fat diet (HFD)

## Abstract

Vascular endothelial cell growth factor A (VEGF-A) signaling promotes the endothelial cell proliferation, macrophage infiltration and foam cell formation, which play pivotal roles in the pathogenesis of atherosclerosis (AS). However, the role of alternative splicing of VEGF here is not known. Here, ApoE (-/-) mice supplied high-fat diet (HFD mice) were used to generate AS, while ApoE (-/-) mice supplied with normal diet (NOR mice) were used as a control. Aortic endothelial cells (AECs) and infiltrated macrophages were purified and quantified by flow cytometry. Alternative splicing of VEGF and the regulator of VEGF splicing, SRPK1, were assessed by RT-qPCR and immunoblotting in both AECs and aortic macrophages. We found that HFD mice developed AS in 12 weeks, while the NOR did not. Compared to NOR mice, HFD mice possessed significantly more AECs and AEC proliferation, and had significantly more aortic infiltrated macrophages and more apoptosis of them. Significant shift of VEGF-A splicing to pro-angiogenic VEGF_165_ was detected in both AECs and macrophages from HFD mice, seemingly through upregulation of SRPK1. In vitro, SRPK1 overexpression significantly increased EC proliferation and macrophage apoptosis. Thus, our data suggest that alternative splicing of VEGF-A to pro-angiogenic VEGF_165_ may contribute to the development of AS.

## Introduction

As the primary cause of heart disease and stroke, atherosclerosis (AS) is characterized with a gradual deposition of lipids and fibrous elements in the arterial wall, due to a chronic inflammatory response to the intramural retention of cholesterol-rich, apolipoprotein B‑containing lipoproteins [1]. Endothelial cell proliferation and macrophage infiltration followed by formation of foam cells hallmark the pathological progression of AS [2].

Vascular endothelial growth factor A (VEGF-A) is the most important mediator of embryonic vascular development and postnatal vessel growth in both physiological and pathological conditions. Although it is well accepted that VEGF-A signaling regulates the endothelial cell proliferation, macrophage infiltration and foam cell formation, all of which play pivotal roles in the AS pathogenesis, the details of the molecular regulation may be complicated due to complexity of the regulation of VEGF-A signaling.

Indeed, VEGF-A exists in several isoforms with strikingly different or even contrasting expression and functions, resulting from alternative splicing of the pro-mRNA transcribed from the 8-exon VEGF-A gene on chromosome [3]. The first discovered VEGF-A isoform is VEGF_165_, which is the most important pro-angiogenic isoform of VEGF-A [4]. Other isoforms including VEGF_121_, VEGF_145_, VEGF_183_, VEGF_189_ and VEGF_206_ [3]. In 2002, VEGF_165b_ was identified as an additional isoform of VEGF-A, which is generated by exon 8 distal splice site selection [5]. The switch between VEGF_165_ and VEGF_165_b has important biological meanings since VEGF_165_ and VEGF_165_b represent pro-angiogenic and anti-angiogenic VEGF-A, respectively [6–8]. Proximal splice site selection in exon 8 of VEGF-A produces pro-angiogenic VEGF_165_, whereas distal splice site selection in exon 8 of VEGF-A generates anti-angiogenic, cytoprotective VEGF_165_b [5]. Moreover, the balance of endogenous pro/anti-angiogenic VEGF-A splice isoforms is regulated by serine/arginine-rich splicing factor protein kinase 1 (SRPK1) [9–11]. SRPK1 phosphorylates serine/arginine-rich splicing factor 1 (SRSF1), resulting in its binding to the VEGF-A mRNA and production of VEGF_165_ [11]. A switch in VEGF-A mRNA splicing to VEGF_165_ has been associated with cancer-associated neovascularization and metastasis [12–14], However a role of alternative splicing of VEGF-A in the pathogenesis of AS is not known.

Apolipoprotein E (ApoE) is a well-known as a strong suppressor for AS, and it functions through regulation of lipoprotein transport and deposit, especially in an inflamed milieu [15]. ApoE-deficient (ApoE -/-) mice display enhanced inflammation in response to hypercholesterolemia and bacterial lipopolysaccharide (LPS) milieu [15]. High fat diet (HFD) induces development of AS in ApoE -/- mice in 12 weeks, which has been used as a model for experimental atherosclerosis [16–18].

In the current study, we addressed the question if alternative splicing of VEGF may play a role in the development of AS. ApoE (-/-) mice supplied HFD (simplified as HFD mice) were used to generate AS, while ApoE (-/-) mice supplied with normal diet (simplified as NOR mice) were used as a control. Aortic endothelial cells (AECs) and infiltrated macrophages were purified by flow cytometry, and analyzed separately for proliferation and apoptosis, respectively. Alternative splicing of VEGF and SRPK1 were analyzed in both AECs and aortic macrophages. The role of SRPK1 and Alternative splicing of VEGF on AEC proliferation and macrophage apoptosis was assessed by overexpression or depletion of SRPK1 in vitro. Our results suggest that alternative splicing of VEGF-A to pro-angiogenic VEGF_165_ may contribute to the development of AS.

## RESULTS

### AS is induced HFD-treated ApoE (-/-) mice

ApoE (-/-) mice were fed with High-fat diet (HFD; simplified as HFD mice) for 12 weeks to induce experimental AS, which was confirmed by increases in plaque area (Figure 1A), by increases in circumferential plaque extension (Figure 1B) and by increases in maximal plaque thickness (Figure 1C), compared to the control littermate ApoE (-/-) mice that had received normal diet (NOR). Thus, HFD induces AS in ApoE (-/-) mice.

**Figure 1:** **AS is induced HFD-treated ApoE (-/-) mice.** ApoE (-/-) mice were fed with High-fat diet (HFD; simplified as HFD mice) for 12 weeks to induce experimental AS. The littermate ApoE (-/-) mice that had received normal diet (NOR) were used as a control. (**A**) Plaque area. (**B**) Circumferential plaque extension. (**C**) Maximal plaque thickness. *p<0.05. N=10.

### AECs increase proliferation and NOS3 expression in AS

Since AEC proliferation is critical for development of AS, we analyzed AECs in this model. First, AECs were purified by flow cytometry, based on CD31, a pan-endothelial cell marker (Figure 2A). We detected more CD31+ AECs in aorta of HFD mice, compared to NOR mice (Figure 2B). BrdU assay was then used to assess the proliferation of AECs. We detected more BrdU+ AECs in HFD mice, compared to NOR mice, shown by representative flow charts (Figure 2C), and by quantification (Figure 2D). CCND1 and CDK4 are two critical factors that promote G0/G1 transition. By Western blotting on the sorted CD31+ AECs, we detected higher CCND1 and CDK4 levels in AECs in HFD mice, compared to NOR mice, shown by representative blots (Figure 2E), and by quantification (Figure 2F-G). Nitric oxide synthase (NOS3) expression in AECs is known to be critical for development of AS. By Western blotting on the sorted CD31+ AECs, we detected higher NOS3 levels in AECs in HFD mice, compared to NOR mice, shown by representative blots (Figure 2E), and by quantification (Figure 2H). Together, these data suggest that AECs increase proliferation and NOS3 expression in AS.

**Figure 2:** **AECs increase proliferation and NOS3 expression in AS.** (**A**-**B**) AECs were purified by flow cytometry, based on CD31, shown by representative flow charts (**A**), and by quantification (**B**). (**C**-**D**) BrdU assay for sorted CD31+ AECs, shown by representative flow charts (**C**), and by quantification (**D**). (**E**) Representative western blots of CD31+ AECs. (**F**-**H**) Quantification of CCND1 (**F**), CDK4 (**G**) and NOS3 (**H**) protein levels in AECs. *p<0.05. N=10.

### Macrophage infiltration and apoptosis increase in AS

Since macrophage infiltration and apoptosis is critical for foam cell formation and development of AS, we analyzed macrophages in this model. First, macrophages were purified by flow cytometry, based on F4/80, a specific macrophage marker (Figure 3A). We detected more F4/80+ macrophages in aorta of HFD mice, compared to NOR mice (Figure 3B). Annexin V assay was then used to assess the apoptosis of macrophages. We detected more apoptotic aortic macrophages in HFD mice, compared to NOR mice, shown by representative flow charts (Figure 3C), and by quantification (Figure 3D). Bcl-2 and cleaved caspase 3 (casps 3) are two critical factors that regulate apoptosis. By Western blotting on the sorted F4/80+ macrophages, we detected lower Bcl-2 and higher casps 3 levels in aortic macrophages in HFD mice, compared to NOR mice, shown by representative blots (Figure 3E), and by quantification (Figure 3F-G). Thus, these data suggest that macrophage infiltration and apoptosis increase in AS.

**Figure 3:** **Macrophage infiltration and apoptosis increase in AS.** (**A**-**B**) Aortic macrophages were purified by flow cytometry, based on F4/80, shown by representative flow charts (**A**), and by quantification (**B**). (**C**-**D**) Annexin V assay for sorted F4/80+ macrophages, shown by representative flow charts (**C**), and by quantification (**D**). (**E**) Representative western blots of F4/80+ macrophages. (**F**-**G**) Quantification of Bcl-2 (**F**) and cleaved caspase 3 (casps 3) (**G**) protein levels in F4/80+ macrophages. *p<0.05. N=10.

### Upregulation of SRPK1 promotes pro-angiogenic splicing of VEGF-A in HFD mice

AS-associated AEC proliferation and macrophage apoptosis are regulated by VEGF-A signaling. However, a role of alternative splicing of VEGF-A in the pathogenesis of AS is not known. Here, we detected a shift of anti-angiogenic splicing of VEGF-A (VEGF_165_b) to pro-angiogenic splicing of VEGF-A (VEGF_165_) in mouse aorta in HFD mice, compared to NOR mice (Figure 4A). Moreover, this shift was detected in both purified AECs and macrophages, at protein levels (Figure 4B-C). SRPK1 is a key promoter of pro-angiogenic splicing of VEGF-A (VEGF_165_), which decreases anti-angiogenic splicing of VEGF-A (VEGF_165_b). We detected increases in SRPK1 mRNA (Figure 4D) and protein (Figure 4E), in both purified AECs and macrophages. These data suggest that upregulation of SRPK1 in HFD mice may promote AEC proliferation and macrophage apoptosis through augmentation of pro-angiogenic splicing of VEGF-A.

**Figure 4:** **Upregulation of SRPK1 promotes pro-angiogenic splicing of VEGF-A in HFD mice.** (**A**) Conventional PCR to show the bands for the anti-angiogenic splicing form of VEGF-A (VEGF_165_b) and the pro-angiogenic splicing form of VEGF-A (VEGF_165_) in mouse aorta. (**B**-**C**) Western blotting for VEGF_165_b and VEGF_165_ in CD31+ AECs and F4/80+ macrophages, shown by representative blots (**B**) and by quantification (**C**). (**D**-**E**) RT-qPCR (**D**) and Western blotting (**E**) for SRPK1 levels in CD31+ AECs and F4/80+ macrophages. *p<0.05. N=10.

### SRPK1 promotes AEC proliferation through increasing pro-angiogenic splicing of VEGF-A in vitro

In order to examine if SRPK1 may promote AEC proliferation through increasing pro-angiogenic splicing of VEGF-A, we generated plasmids carrying SRPK1 or shSRPK1, which overexpress or inhibit expression of SRPK1. A plasmid carrying a scramble sequence (SCR) was used as a control. These plasmids were used to transfect a mouse endothelial cell line, MS1. The RT-qPCR for SRPK1 levels in the transfected MS1 cells was done to confirm the overexpression or depletion of SRPK1 in the MS1 cells (Figure 5A). The protein levels were determined, showing that overexpression of SRPK1 in MS1 cells significantly increased the ratio of VEGF_165_ to VEGF_165_b, the levels of CCND1, CDK4 and NOS3, shown by representative blots (Figure 5B), and by quantification (Figure 5C-F). On the other hand, depletion of SRPK1 significantly decreased the ratio of VEGF_165_ to VEGF_165_b, the levels of CCND1, CDK4 and NOS3, shown by representative blots (Figure 5C), and by quantification (Figure 5C-F). Tube formation assay was applied using these SRPK1-modified MS1 cells, showing that overexpression of SRPK1 significantly increased tube formation while depletion of SRPK1 significantly decreased tube formation in MS1 cells (Figure 5G-H). In order to confirm whether SRPK1 works through VEGF_165_/VEGF_165_b to affect tube formation, co-transfection shSRPK1 with VEGF_165_, or co-transfection SRPK1 with VEGF_165_b were performed. We found that VEGF_165_ significantly attenuated the effects of shSPRK1 on tube formation, and VEGF_165_b significantly attenuated the effects of SPRK1 on tube formation, suggesting that SRPK1 works through VEGF_165_/VEGF_165_b to affect tube formation (Figure 5G-H). Together, these data suggest that SRPK1 may promote AEC proliferation through increasing pro-angiogenic splicing of VEGF-A in vitro.

**Figure 5:** **SRPK1 promotes AEC proliferation through increasing pro-angiogenic splicing of VEGF-A in vitro.** (**A**) RT-qPCR for SRPK1 in shSRPK1, or SCR, or SRPK1- transfected MS1 cells. (**B**) Representative western blots of SRPK1-modified MS1 cells. (**C**-**F**) Quantification of ratio of VEGF_165_ versus VEGF_165_b (**C**), CCND1 (**D**), CDK4 (**E**) and NOS3 (**F**) protein levels in SRPK1-modified MS1 cells. (**G**-**H**) Tube formation assay using SRPK1/VEGF_165_/VEGF_165_b -modified MS1 cells, shown by representative images (**G**), and by quantification (**H**). *p<0.05. N=5. Scale bars are 50µm.

### SRPK1 promotes macrophage apoptosis through increasing pro-angiogenic splicing of VEGF-A in vitro

In order to examine if SRPK1 may promote macrophage apoptosis through increasing pro-angiogenic splicing of VEGF-A, we used the generated SRPK1-modifying plasmids to transfect a mouse macrophage line, RAW264.7. The RT-qPCR for SRPK1 levels in the transfected RAW264.7 cells was done to confirm the overexpression or depletion of SRPK1 in the RAW264.7 cells (Figure 6A). The protein levels were determined, showing that overexpression of SRPK1 in RAW264.7 cells significantly increased the ratio of VEGF_165_ to VEGF_165_b, the levels of casps 3, and decreased the levels of Bcl-2, shown by representative blots (Figure 6B), and by quantification (Figure 6C-E). On the other hand, depletion of SRPK1 significantly decreased the ratio of VEGF_165_ to VEGF_165_b, the levels of casps 3, and increased the levels of Bcl-2, shown by representative blots (Figure 6B), and by quantification (Figure 6C-E). Annexin V assay was applied using these SRPK1-modified RAW264.7 cells, showing that overexpression of SRPK1 significantly increased apoptosis while depletion of SRPK1 significantly decreased apoptosis in RAW264.7 cells (Figure 6F-G). In order to confirm whether SRPK1 works through VEGF_165_/VEGF_165_b to affect macrophage apoptosis, co-transfection shSRPK1 with VEGF_165_, or co-transfection SRPK1 with VEGF_165_b were performed. We found that VEGF_165_ significantly attenuated the effects of shSPRK1 on macrophage apoptosis, and VEGF_165_b significantly attenuated the effects of SPRK1 on macrophage apoptosis, suggesting that SRPK1 works through VEGF_165_/VEGF_165_b to affect macrophage apoptosis (Figure 6F-G). Together, these data suggest that SRPK1 may promote macrophage apoptosis through increasing pro-angiogenic splicing of VEGF-A in vitro. The findings in the current study were then summarized in a schematic, showing that SRPK1-mediated alternative splicing of VEGF-A to pro-angiogenic VEGF_165_ may contribute to the development of AS, possibly through increasing AEC proliferation and macrophage apoptosis (Figure 7).

**Figure 6:** **SRPK1 promotes macrophage apoptosis through increasing pro-angiogenic splicing of VEGF-A in vitro.** (**A**) RT-qPCR for SRPK1 in shSRPK1, or SCR, or SRPK1- transfected RAW264.7 cells. (**B**) Representative western blots of SRPK1-modified RAW264.7 cells. (**C**-**E**) Quantification of ratio of VEGF_165_ versus VEGF_165_b (**C**), Bcl-2 (**D**) and Casps 3 (**E**) protein levels in SRPK1-modified RAW264.7 cells. (**F**-**G**) Annexin V assay for SRPK1/VEGF_165_ /VEGF_165_b -modified RAW264.7 cells, shown by quantification (**F**), and by representative flow charts (**G**). *p<0.05. N=5. Scale bars are 50µm.

**Figure 7:** **Schematic of the model.** SRPK1-mediated alternative splicing of VEGF-A to pro-angiogenic VEGF_165_ may contribute to the development of AS, possibly through increasing AEC proliferation and macrophage apoptosis.

## DISCUSSION

A well-coordinated immune-inflammatory interaction among endothelial cells, macrophages and smooth muscle cells controls the development of AS. Specifically, high blood sugar is a potent pro-atherosclerotic factor capable to induce experimental AS, pronounced in ApoE (-/-) mice [16–18].

Angiogenesis occurs in concurrence with development of AS [19–21], while the exact role of angiogenesis in AS is not completely understood. Although suppression of intimal angiogenesis in ApoE (-/-) mice has been shown to reduce AS [22], the exact role of VEGF-A in this study is not certainly validated. Indeed, the exact specification of VEGF signaling includes determination of the involvement of different VEGF family members, e.g. VEGF-A, VEGF-B, VEGF-C, VEGF-D, VEGF-E and placental growth factor (PlGF) [23]. Moreover, alternative splicing of VEGF-A mRNA to result in different isoforms with distinct functions further increases the complexity of VEGF signaling. Indeed, the molecular control of C’-terminal splice site to decide the balance between pro-angiogenic and anti-angiogenic VEGF-A has been shown to a very important regulator of VEGF-A activity, since it has been shown that the basal expression of VEGF-A is dominated by the VEGF_165_b isoform in most tissues in adults [24]. Interestingly, only the placenta, the only known tissue with active angiogenesis, expresses less the VEGF_165_b isoform than the VEGF_165_ isoform [24]. Thus, it is compelling to study the alternative VEGF splicing in the setting of AS.

In the current study, we not only detected the increases of the ratio of VEGF_165_ versus VEGF_165_b in both AECs and macrophages, but also found that this changes in VEGF-A mRNA splicing should result from upregulation of its regulator, SRPK1. SRPK1 is a serine/arginine-rich kinase which phosphorylates specific substrates at serine residues located in regions rich in RS domains to mediate phosphorylation of SR splicing factors to control the events of alternative mRNA splicing.

Recently, Batson et al. showed that SRPK1 regulates alternative splicing of VEGF-A to pro-angiogenic isoforms and specific inhibitors occupy a binding pocket created by the unique helical insert of SRPK1 to selectively suppress SRPK1 kinase activity, resulting in potent abortion of blood vessel growth in mouse models of choroidal angiogenesis [25]. Here, in either a loss-of-function experiment using shSRPK1 or a gain-of-function experiment using SRPK1, we found that in both macrophages and endothelial cells, SRPK1 induced alternative VEGF-A splicing into a pro-angiogenic VEGF_165_ isoform. The outcome of this augmentation in pro-angiogenic VEGF-A, resulting in increases in cell proliferation in AECs and enhanced angiogenesis, and increases in macrophage apoptosis to enhance foam cell formation. Since SRPK1 may have many splice factors as substrates and these splice factors could control splicing of genes other than VEGF-A, we added additional experimental conditions (co-transfection shSRPK1 with VEGF_165_, or co-transfection SRPK1 with VEGF_165_b to show that indeed VEGF splicing is the main connection between elevated SRPK1 and AS-associated phenomena on AEC proliferation and macrophage apoptosis.

Moreover, NOS3 is a well-known factor that increases its expression in endothelial cells in AS. NOS3 induces significant vasodilatation that contributes the development of AS [26]. Hence, the SRPK1-induced alternative VEGF-A to favor formation of pro-angiogenic VEGF_165_ seems to promote AS formation via all effects on AECs and macrophages.

It may be interesting to study the regulation of SRPK1 in HFD mice, which may help to identify novel targets to prevent the development of AS. Moreover, in vivo interference with SRPK1 expression may be interesting to be performed to identify the direct effects of SRPK1 activity on AS development.

## MATERIALS AND METHODS

### Ethics, consent and permissions

The study was approved by the Animal Care and Use Committee of Shanghai Jiao Tong University. All experimental procedures were performed according to “Guide for the Care and Use of Laboratory Animals”, an US National Institutes of Health press.

### AS model in mice

ApoE (−/−) mice were originally purchased from Jackson Laboratory (Bar Harbor, ME, USA) and bred in-house under sterile animal room conditions (22 ± 2°C; 55–60% humidity). Twenty female animals of 10 weeks of age were randomly divided into two groups: the normal-diet group (NOR) and the high-fat diet (HFD) group for the respective diet for 12 weeks.

The aortic roots were dissected out for histology or digestion into single cells followed by flow cytometry-based cell purification. For histology, the tissue was fixed with 4% paraformaldehyde for 6 hours, cryo-protected in 30% sucrose for 12 hours, and then embedded in OCT. Cross-section was done in 5μm thickness. Atherosclerotic lesions of the aortic root were assessed based on every 5^th^ slide from thirty serial sections in between the aortic root to the midportion of descending thoracic aorta. Slides were stained with Verhoeff reagent and counterstained with hematoxylin. Plaque area was measured as the difference between lumen area and the area delimited by the internal elastic lamina, normalized to total vessel cross-sectional area. Plaque circumferential extension was determined by the ratio of the cross-sectional circumferential length of each plaque to total luminal circumference. The maximum thickness of the plaque for each section was finally determined. Quantification of the images was measured using NIH ImageJ software (Bethesda, MD, USA).

### Flow cytometry-based cell purification and analysis

The tissue was dissociated into single cells by incubation with Accutase Enzyme Cell Detachment Medium (Thermo Fisher Scientific Inc., Waltham, MA, USA), according to the instruction from the manufacturer. For isolation of endothelial cells or macrophages, the single cell tissue cells were incubated with PEcy7-conjugated anti-CD31 antibody, or APC-conjugated anti-F4/80 antibody, respectively (Becton-Dickinson Biosciences, San Jose, CA, USA). BrdU assay was done with a bromodeoxyuridine (BrdU) flow kit (Becton-Dickinson Biosciences). A FITC Annexin V Apoptosis Detection Kit I (Becton-Dickinson Biosciences) was used to analyze apoptosis of the cells, in which a double staining with FITC-Annexin V and propidium iodide (PI) is required. Analysis and cell sorting were performed using FACScan flow cytometer (Becton-Dickinson Biosciences) and Flowjo software (Flowjo LLC, Ashland, OR, USA).

### Transfection of cells in vitro

A mouse endothelial cell line, MS1, and a mouse macrophage cell line, RAW264.7, are both purchases form American Type Culture Collection (ATCC, Rockville, MD, USA). Both lines were cultured in DMEM media (Invitrogen, CA, Carlsbad, USA) supplied with endothelial cell growth factors, 5% fetal bovine serum (FBS, Invitrogen) and 1% penicillin/streptomycin (Invitrogen). Cells were kept at 37°C with 5% CO_2_. MS1 and RAW264.7 were transfected with SRPK1 or short hairpin small interfering RNA for SRPK1 (shSRPK1; a 50%-to-50% mixture of 2 sequences: 5’-UUAAUGACUUCAAUCACUCCAUUGC-3’ and 5’-UAAGAAAUCUGUGAAGCCAGCUGCC-3’), or a scramble control (SCR) (RiboBio Co., Ltd., Guangzhou, Guangdong, China), or VEGF_165_, or VEGF_165_b, using Lipofectamine 3000 reagent (Invitrogen), according to the manufacturer's instructions. The transfection efficiency at a multiplicity of infection of 100 was nearly 100% without noticeable cell death.

### RNA extraction, conventional PCR and RT-qPCR

Total RNA was extracted with RNeasy mini kit (Qiagen, Hilden, Germany). Complementary DNA (cDNA) was randomly primed from 2μg of total RNA using High-Capacity cDNA Reverse Transcription Kit (Applied Biosystems, Foster City, CA, USA). Conventional PCR for determining proximal and distal splice forms of VEGF-A used the following primer sets (5’-GGCAGCTTGAGTTAAACGAAC-3’ and 5’-ATGGATCCGTATCAGTCTTTCCTGG-3’). The reaction was 30 cycles with denaturing at 95 °C for 60 s, annealing at 55 °C for 60 s, and extending at 72 °C for 60 s. This reaction usually resulted in one amplicon of 130bp (VEGF_165_) and one amplicon of 64bp (VEGF_165_b). RT-qPCR was performed in duplicate with QuantiTect SYBR Green PCR Kit (Qiagen). All primers were purchased from Qiagen. Data were collected and analyzed using 2-△△Ct method for quantification. RT-qPCR values were presented as relative values, which was obtained after sequential normalization against α-tubulin and the experimental controls.

### Western blotting

Lysis was done with RIPA buffer (Sigma-Aldrich, St. Louis, MO, USA) containing protease and phosphatase inhibitors (Complete ULTRA Tablets, Roche, Nutley, NJ, USA). After centrifugation, the supernatant was collected and quantified by BCA assay (Sigma-Aldrich). The proteins were then separated by SDS-PAGE and transferred to nitrocellulose membranes. After blocking with 5% non-fat milk, the membranes were probed with rabbit anti-VEGF_165_ (R&D System, Los Angeles, CA, USA), rabbit anti- VEGF_165_b (R&D System), rabbit anti-SRPK1 (Cell Signaling Technology, Danvers, MA, USA), anti-Bcl-2 (Cell Signaling Technology), rabbit anti-cleaved caspase 3 (casps3; Cell Signaling Technology), rabbit anti-CCND1 (Santa Cruz Biotechnology, Dallas, Texas, USA), rabbit anti-CDK4 (Santa Cruz Biotechnology), rabbit anti-nitric oxide synthase (anti-NOS3; Cell Signaling Technology), and rabbit anti-α-tubulin (Cell Signaling Technology, Danvers, MA, USA). Secondary antibodies are HRP-conjugated against rat or rabbit (Jackson ImmunoResearch Labs, West Grove, PA, USA). The protein levels were first normalized to α-tubulin, and then normalized to the experimental controls. Densitometry of Western blots was quantified with NIH ImageJ software.

### Tube formation assay

The genetically modified MS1 cells were embedded in a collagen gel, and plated on a culture plate. The plate was returned to the CO_2_ incubator. Media was replenished every day, and culture images were taken after 3 days.

### Statistical analysis

The data was statistically analyzed with GraphPad Prism (version 7, GraphPad Software, Inc. La Jolla, CA, USA). All values are depicted as mean ± standard deviation of the mean. All data were statistically analyzed by one-way ANOVA with a Bonferroni correction, followed by Fisher's exact test to compare 2 groups. Significance was considered when p < 0.05.

### Declarations

Availability of data and material: All data generated or analyzed during this study are included in this published article.

## CONCLUSIONS

To summarize, here we provide evidence to show that SRPK1-mediated alternative splicing of VEGF-A to pro-angiogenic VEGF_165_ may contribute to the development of AS, possibly through increasing AEC proliferation and macrophage apoptosis.

## Supplementary Material

Supplementary Figures
